This article has been retracted.

# Analysis of the Effect of Intensive Care Based on Lean Nursing Intervention

**DOI:** 10.1155/2021/7805124

**Published:** 2021-09-29

**Authors:** Jing Yang, Mingjun Xu, Yili Wang, Zhiqiang Gao

**Affiliations:** First Affiliated Hospital of Gannan Medical University, Ganzhou, China

## Abstract

In order to improve the effect of intensive care, this paper proposes a lean nursing intervention method and evaluates the lean nursing intervention through a controlled experiment. According to the actual situation of intensive care, this paper starts with the research from several aspects of patients' ICU nursing time, patients' satisfaction, patients' pathological knowledge familiarity, patients' autonomous nursing, and enthusiasm of patients and their families. Moreover, this paper collects and displays experimental results through mathematical statistics, gives patients lean management concepts and methods based on routine care, and finds that it has good management effects. Thus, lean management concepts and methods can effectively improve the anxiety state of critically ill patients, improve the patient's knowledge of disease, and reduce adverse nursing events to improve patient nursing satisfaction, which is worthy of further promotion in the clinic.

## 1. Introduction

Intensive care is a specialised nursing field with acute and critically ill patients as the main service target [1]. The intensive care unit is important for centralized monitoring, intensive treatment, and continuous care of patients with acute and critical illness [2]. ICU nurses must have advanced theoretical knowledge and abilities, be competent in using a variety of sophisticated tools and equipment, and correctly evaluate and respond to complicated and hazardous changes in the patient's condition. Furthermore, they play a vital role in the rescue and monitoring of critically sick patients [3]. With the rapid rise of intensive care medicine and the extensive establishment of intensive care units, intensive care practice has also been given higher requirements and updated connotations.

The intensive care unit for intensive care, also known as the comprehensive treatment room of the intensive care unit, gathers critically ill patients and provides the best protection in terms of manpower, material resources, and technology. At the same time, when the patient is not accompanied by family members and faces the critical and complex condition alone, the unknown recovery from the disease, and even the threat of death, the patient is prone to negative emotions such as anxiety/depression, which aggravates the patient's condition and is not conducive to the long-term prognosis of the patient. Past studies have shown that ICU patients' disease progresses rapidly and their families lack understanding of the disease. Therefore, ICU family members hope to understand the patient's disease outcome through various methods. Medical personnel at the critical care unit, on the other hand, work at a rapid pace and with high workloads, and family members have limited access to information due to the intensive care unit's tight management. Family members of sober ICU patients are particularly affected by this tendency [4].

The intensive care unit/ward is a comprehensive department accepting and treating critically ill and emergency patients. Moreover, it is a department that concentrates the high-precision technical equipment and personnel of the hospital, and it has more advanced medical equipment and can continuously monitor the vital signs after major operations, as well as in emergency and critical patients. All kinds of unfamiliar instruments and equipment, such as electrocardiogram monitors and ventilators, are piled around ICU patients. Noisy sound stimulation, such as ventilator sound and light alarms, damaging pressure drainage equipment, and ECG monitoring equipment, as well as pain from disease or postoperative traumatic stimulation, cause ICU patients to remain fearful, sleepless, in pain, and under mental and psychological stress in the absence of family members. It is precisely because of this that, in the special environment of the ICU ward, although advanced treatment and rescue are provided for patients, at the same time, compared with the general ward, ICU patients are under tremendous mental pressure. ICU patients have to endure the pain caused by illness and medical trauma and endure the psychological and spiritual trauma caused by isolation from their loved ones. ICU patients mainly include patients with severe or multiple injuries that require functional support and functional status monitoring, patients with severe metabolic disorders or acute metabolic disorders, patients with severe surgical trauma who need life support and monitoring, patients with life-threatening complications such as hemorrhage after surgery, patients with acute heart failure, renal failure, and other organs with acute dysfunction or failure, patients with severe infections, and patients after organ transplantation. The abovementioned severe or acute diseases have caused severe physical and psychological trauma to ICU patients, causing many ICU patients to experience unhealthy or negative emotions such as tension, fear, and depression. At the same time, patients may even experience some abnormal behaviors and cognitive decline, such as confusion, nonsense, and insomnia. In addition, such patients are often more prone to anger and conflicts with family members and medical staff. Moreover, these bad moods, sleep disorders, fear and tension, etc. often lead to a decrease in the immunity of ICU patients, thereby prolonging the recovery time of their own diseases and even aggravating the risk of the patient's condition. Therefore, it is urgent to explore the factors that can cause patients' psychological and mental disorders in the ICU environment to improve the nursing methods of ICU patients. At the same time, various risk factors need to be reasonably controlled to reduce the psychological and mental disorders of ICU patients and promote the treatment and recovery of patients.

This paper combines lean nursing intervention methods to formulate intensive care methods and combines experimental research to explore the intensive care effects of lean nursing interventions.

### 1.1. Related Work

In view of the particularity of the intensive care specialty, foreign countries attach great importance to the standardization and development of intensive care practice. Some developed countries and regions have long established intensive care professional organizations and formulated and published a series of industry standards and practice guidelines on intensive care practice activities, professional skills of ICU nurses, and critical care job models. These industry standards and practice guidelines are based on sound science and practice, provide valuable clinical advice, and help to advance and improve the quality of critical care and the professional skills of ICU nurses. The United States presently has the most developed and comprehensive intensive care practice of any nation. In the 1990s, the American Critical Care Association developed a collaborative model to guide the standardization and development of critical care practice in the country based on the physical and psychological needs of critically ill patients throughout the medical process and the fit with ICU nurses and the medical environment. The core idea of this theoretical model is that the characteristics and needs of critically ill patients and their families influence and determine the characteristics and ability requirements of ICU nurses. When the professional ability of ICU nurses matches the medical needs of critically ill patients, the best nursing care and the best clinical outcome will be achieved [5]. According to the characteristics and needs of critically ill patients and their families, the American Academy of Critical Care has proposed 8 professional abilities that ICU nurses should possess in a collaborative model. They are clinical judgment ability, nursing practice ability, support and moral endorsement ability, collaboration ability, system thinking ability, ability to respond to diversity, ability to promote learning, and ability to clinical inquiry [6]. After that, the American Critical Care Association developed specific behavioral descriptions of various professional abilities of ICU nurses through investigation and research on critical care practice. Moreover, according to these specific behavior descriptions, each professional ability is divided from low to high into three competence levels: level 1, level 3, and level 5, which represent the three practical levels of novice, competitive, and expert [7]. The American Academy of Critical Care has constantly updated and enhanced the collaborative model in order to better support the standardization and growth of intensive care practice and intensive care advanced care practice. Furthermore, it employs the collaborative model as the theoretical framework for developing professional competence requirements for ICU nurses of various levels and subdivisions, such as intensive care specialist nurses, intensive care senior practice nurses, and cardiology specialist intensive care nurses, as well as specialised practice activities and advanced practice activities that are related to the collaborative model. Moreover, taking into account the rapid development and changes of intensive care practice, the American Critical Care Association conducts investigations and studies on current intensive care practice every 3–5 years. At the same time, it constantly revises, updates, and perfects the collaborative model based on the survey results [8] to ensure that the industry standards and practice guidelines of critical care practice can match the rapidly expanding new knowledge and new technologies. For more than 20 years, the collaborative model of the American Academy of Intensive Care has been praised and recognized by many intensive care professional organizations and intensive care nurses. Moreover, it is widely used in intensive care clinical practice [9], intensive care education [10], the establishment of advanced practice models of intensive care [11], ICU nurse professional competence training [12], and many other fields. At the same time, many countries and regions refer to and learn from the collaborative model of the American Institute of Intensive Care and the survey and research of the current situation of critical care practice to draft, design, and revise industry standards and practice guidelines that are in line with their own country and region's critical care practice [13]. In order to standardize and promote the development of intensive care practice, the Hong Kong Society of Intensive Care has formulated the intensive care practice standards and the intensive care advanced practice nurse competency framework [12]. The British Ministry of Health and the British Institute of Intensive Care have issued a series of industry standards and practice guidelines on intensive care practice and intensive care advanced care practice. It aims to help clinical nurses and nursing managers make correct clinical decisions and promote safe intensive care practices [14].

## 2. Research Methods

We selected the postoperative patients with femoral shaft fractures admitted to the ICU of a hospital from June 2018 to June 2021 as the research object.

Inclusion conditions: (1) after unilateral femoral shaft fracture, head CT and M arsenic examination confirmed that there was no severe brain injury; (2) the patient is in stable condition, has a clear consciousness, and has no history of mental illness and severe cognitive dysfunction, but needs intensive monitoring, and the APACHE II score is 5–25; (3) the ICU hospital stay is ≥5 days, and age is 18–75 years; (4) the patient has no cognitive impairment and can complete the questionnaire survey autonomously or with the cooperation of family members; and (5) the patient and family members have informed consent and are willing to cooperate in the research.

ICU patients with femoral shaft fractures who met the inclusion criteria were assigned to the intervention group and the control group according to the odd and even numbers. According to the order of admission to the ICU, the first one was assigned to the intervention group, the second was assigned to the control group, and so on, and the two groups were separated from each other to avoid the contaminated effect of the two groups of patients [15].

The control group used ICU routine nursing: (1) all patients are required to continue ECG monitoring for 24 hours, measuring and recording heart rate (aiR), blood oxygen saturation (SpO_2_), and respiratory rate (heart and blood pressure (BP) every hour. Moreover, the patient's body temperature is measured every 4 hours and recorded once. For patients newly transferred to ICU ward, different vital signs must be measured and recorded in real time. Then monitor the changes of patients' health in real time and provide professional medical treatment for them. When an ICU patient arrives on the ward, the nurse must assist the patient in becoming acquainted with the surroundings as quickly as possible, as well as getting to know the appropriate nursing staff and actively assisting the patient in formulating a daily diet. At the same time, it is necessary to understand the patient's psychological state through familiarity and face-to-face communication with the patient's clinical condition and social background, family environment, academic background, and other materials and patiently answer patients' questions. Moreover, it is necessary to untie the patient's heart knot in conversation, help the patient adapt to the role, correct the attitude, and eliminate bad emotions to cooperate with clinical treatment and nursing work actively. Keeping the intensive care unit clean and quiet is necessary, and the indoor temperature is suitable (25–27°C). At the same time, it is necessary to keep the light in the ward soft, avoid too dark light to affect the mood of the patient, and ensure regular ventilation to maintain air circulation. In addition, lunch breaks and nights require gentle and skilled nursing activities. (2) Disease and pain management: it is important to identify the location and type of the patient's pain as soon as possible and to report it to the responsible physician. Furthermore, in order to relieve the patient's pain, it is essential to follow the doctor's recommendation for therapy or medicine while under the supervision of a doctor. Simultaneously, sedative and analgesic medicines must be used as needed to relieve pain and suffering and assist patients in falling asleep, and it is necessary to educate patients about the effectiveness and risks of the drugs, standardize drug usage, and prevent accidents. In addition, it is necessary to guide the patient to move correctly according to the clinical condition to improve the patient's physical and psychological state. (3) It is necessary to follow the doctor's order to plan the infusion strictly, all drugs must be checked 3 times and confirmed 7 times, and the patient's 24 h liquid intake and output must be accurately recorded, and an infusion pump can be used when necessary. (4) Pressure ulcer scores, sedation scores, and GCS scores must be implemented in time to prevent pressure ulcers. At the same time, it is necessary to do morning and evening care, perineal scrubbing, and oral care to make the critically ill patient comfortable. Teaching imitation: for conscious patients, nurses are required to teach the patients to master some simple operation methods, such as turning over, expectoration, coughing, and early bed function training. (5) It is necessary to strictly implement the handover work and earnestly implement the corresponding handover responsibilities of each shift. (6) Central venous catheters, tracheal intubation, tracheotomy, and mechanical ventilation must all be managed. (7) It is critical to maintain the drainage tube, urine tube, and other pipes clear in order to avoid tube loss and blockage, as well as cross-infection. (8) Psychological counseling: it is necessary to provide psychological counseling and comfort, strive for the cooperation of the social coupling system, and do well in nursing measures such as knowledge propaganda and education. It is necessary to improve the family communication process, through the family to understand the patient's social role, family members, degree of concern for the disease, cognition, and economic conditions. At the same time, it is necessary to carry out the “five steps” of bedside communication, narrow the distance with the patient, and give the patient emotional support. Nurses can judge the information they want to express through the patient's gestures and facial expressions, or write simple words on their hands or on paper to communicate for some patients who are unable to communicate in language but are conscious, such as patients receiving ventilator-assisted treatment, tracheal intubation, and so on. (9) The specific contents of health education are as follows: (1) oral explanation: language explanation is the most important and basic way of education; (2) patient questions: patients need to be encouraged to ask questions and nurses should answer patiently. At the same time, it is necessary to pay attention to the two-way nature of health education and the communication of educational information [16].

The intervention group adds comprehensive and lean nursing methods based on ICU routine nursing.

(1) Form a lean management group: the Orthopedics Lean Management Team was established by the orthopaedics department's chief nurse, who also acted as the team leader, under the direction of the Nursing Department. Other orthopedic nurses were enlisted as team members, and two experienced senior nurses from the department were chosen to serve as deputy team leaders. Before the application of the lean management model, the team leader held a discussion meeting to brainstorm and summarize the inadequate links and redundant links in the past nursing management, read the literature, and comb the recent research results and the actual situation in orthopedic nursing management to sort out the problems. Put forward optimization opinions and form an effective set of optimized nursing management plans and nursing operation procedures. After implementing the lean management plan, the group regularly organizes seminars to reflect on and discuss the problems in the implementation process and dynamically adjust the plan according to the actual situation [17]. (2) Strengthen nursing training: 121 nursing skills are the cornerstone of orthopedic care. Only good nursing skills can help patients recover their mobility as soon as possible, which is why senior nurses often gain the trust of patients. After implementing the lean management model, regular nursing skills training is carried out in the department, and assessments are arranged after the training is completed. Those who do not meet the assessment standards need to strengthen skills training further. Also, the lean management team conducts surprise spot checks on nursing skills to urge the department nurses to learn actively and make continuous progress. (3) Standardize process management: optimize the flow of patients from the hospital to discharge. A simple and effective flow can improve the patient's medical experience. A designated individual will be in charge of welcoming the patient once they have been admitted to the hospital. He will introduce the ward environment of the undergraduate room and related precautions to the patient in a patient and kind manner, as well as explain the patient's knowledge of the disease, treatment plan, and prognosis to the patient and their family members, in order to improve the patient's medical treatment confidence. Strengthen nurse care throughout the perioperative phase and respond to patients' and families' concerns. Nurses must improve perioperative ward inspections, closely monitor the patient's vital signs, and immediately notify the doctor when the patient's health deteriorates so that the patient's life is not jeopardised. Nurses are required to participate in bedside handover shifts. The responsible nurse must understand the patient's condition and organize general nurse rounds once a week. The leader or deputy leader of the lean management team will conduct spot checks, comments and questions, and urge the undergraduate nurses to be more active and pay attention to the patient's condition. Before the patient is discharged from the hospital, a special person will be arranged to explain the precautions after discharge to the patient and family members, and the patient is asked to review regularly, strengthen functional exercise, and cooperate with the follow-up [18]. (4) Carry out nursing lectures: regularly hold lectures on orthopedic nursing knowledge and take turns to give lectures by general nurses. The lectures are conducted in the form of PPT or case discussions. The content of the lectures can include recent nursing research, knowledge of orthopedic functional exercises, and related knowledge of health education. Patients and their families are invited to participate in the lectures and provide valuable suggestions. Department nurses may benefit from knowledge lectures by improving their theoretical knowledge, learning new nursing methods, and providing better nursing care to patients. (5) Make flexible scheduling a priority: currently, orthopedic nurses have a lot of work to do, and the high physical and mental stress makes it difficult to provide high-quality nursing care. The flexible scheduling system is conducive to alleviating the physical and mental pressure of nurses. In the case of ensuring the nursing strength and staffing of the departments, a flexible shift scheduling system is implemented, shifts are adjusted according to the requirements of nurses, and nurses are reasonably arranged to rest, thereby improving the quality of nursing [19].

*Evaluation Indicators*. According to the actual situation of intensive care, this paper conducts research from several aspects of patients' ICU nursing time, patients' satisfaction, patients' pathological knowledge familiarity, patients' autonomous nursing, and enthusiasm of patients and their families.

## 3. Results

The test results are clearly displayed in this paper using statistical tables and graphs. The control group is represented by the yellow curve in the statistical diagram, whereas the blue curve represents the test group. This study tracks the patient's ICU nursing time, which is primarily the time it takes for the patient to transition from severe to mild condition.  Table 1 and Figure 1 show the statistical time of the test group and the control group.

As can be seen from the statistical analysis above, lean nursing approaches can successfully minimize the time spent in critical care and increase patient recovery. Furthermore, the test group recovered faster than the control group. The patient's happiness is next measured, and the findings are given in Table 2 and Figure 2.

The lean nursing intervention proposed in this paper can play a good effect in intensive care from the above statistical results. Furthermore, compared with the control group, the test group patients have higher satisfaction. On this basis, the patient's pathological knowledge familiarity is tested, and the results obtained are shown in Table 3 and Figure 3.

According to the findings, patients in the test group are more familiar with pathological knowledge than the control group. As a result, lean nursing intervention can assist patients in comprehending pathogenic knowledge, resulting in a better auxiliary effect on rehabilitation follow-up. We conduct statistics on the effect of patients' autonomous nursing on this premise, and the findings are displayed in Table 4 and Figure 4.

The patients in the test group have a certain autonomous nursing ability based on the propaganda of pathological information and nursing knowledge of lean nursing, as shown in the above research results. Following that, the patients' and their families' enthusiasm is assessed, with the results displayed in Table 5 and Figure 5.

It can be seen from the above research that the lean nursing intervention proposed in this paper can play an important role in intensive care and help patients and their families to improve their enthusiasm for treating diseases.

The rate of disease knowledge mastery in the lean group was significantly higher than that in the conventional group.

## 4. Conclusion

The condition of critically ill patients is more critical and complex, and nursing risks exist in every link of patient treatment, nursing, and examination. Once an adverse nursing event occurs, it will affect the smooth treatment of patients and easily cause nurse-patient disputes. Lean management concept is a management concept that creates as much value as possible with minimal investment in resources. It has been gradually applied to nursing management and has the effect of improving the quality of nursing. The application of lean management concepts in the process of patient care management can effectively release unnecessary steps and resources in nursing work, making nursing work more targeted and effective, so that patients receive better quality, more professional, and more intimate nursing services. In this regard, this study gives patients lean management concepts and methods on the basis of routine nursing and found that it has good management effects. Lean management concepts and methods can effectively improve the anxiety state of critically ill patients, improve the patient's knowledge of disease, and reduce good nursing incidents, thereby increasing the patient's nursing satisfaction, which is worthy of further clinical promotion.

## Figures and Tables

**Figure 1:** Line chart of ICU nursing time of critically ill patients.

**Figure 2:** Line chart of satisfaction after nursing for critically ill patients.

**Figure 3:** Line chart of familiarity of patients' pathological knowledge.

**Figure 4:** Line chart of the effect of patients' autonomous nursing.

**Figure 5:** Line chart of enthusiasm of patients and their families.

**Table 1:** Statistical results of ICU nursing time of critically ill patients.

No.	Control group (D)	Test group (D)
1	9.0	10.8
2	10.6	7.5
3	13.9	8.6
4	9.8	10.1
5	14.2	10.7
6	14.7	7.3
7	11.2	7.5
8	11.0	8.1
9	14.7	9.4
10	12.5	10.9
11	10.1	11.8
12	11.6	9.3
13	9.6	8.2
14	13.3	8.8
15	14.9	10.4
16	12.8	10.2
17	14.5	7.4
18	13.3	10.2
19	14.1	7.3
20	11.3	11.5
21	10.4	9.2
22	13.1	11.4
23	14.9	9.4
24	12.0	9.6
25	12.9	9.0
26	14.7	12.0
27	13.3	9.0
28	13.9	11.2
29	9.5	7.7
30	13.2	11.8
31	11.9	11.3
32	12.7	10.2
33	11.4	11.0
34	11.5	8.6
35	9.1	8.6
36	15.0	9.8
37	12.8	9.5
38	9.3	10.6
39	9.6	7.2
40	10.2	8.0
41	12.3	11.6
42	11.7	9.0
43	9.4	10.0
44	10.2	10.1
45	11.7	9.7
46	10.4	11.3
47	11.3	9.3
48	12.1	7.9
49	13.7	8.4
50	10.1	8.8
51	9.9	9.2

**Table 2:** Statistical table of satisfaction of critically ill patients after nursing.

No.	Control group	Test group
1	90.09	79.45
2	91.86	88.61
3	86.81	92.53
4	73.33	97.08
5	86.62	93.36
6	87.16	83.90
7	84.59	97.14
8	81.80	89.90
9	80.34	96.05
10	78.86	81.84
11	78.87	92.11
12	78.00	80.44
13	88.54	88.05
14	80.34	91.14
15	84.31	96.98
16	75.02	89.08
17	81.64	92.71
18	73.81	96.41
19	89.59	97.72
20	86.68	92.59
21	91.10	79.69
22	91.85	85.74
23	84.92	84.29
24	71.72	89.39
25	91.69	82.30
26	80.23	83.94
27	88.12	88.87
28	73.44	97.98
29	73.01	79.36
30	82.83	94.33
31	90.74	90.22
32	86.89	86.21
33	86.62	82.93
34	81.26	80.21
35	71.63	90.09
36	85.47	84.91
37	87.73	83.98
38	74.98	83.09
39	90.08	94.62
40	78.21	84.87
41	91.08	92.79
42	79.43	87.64
43	76.30	96.60
44	90.55	91.70
45	76.98	92.91
46	85.64	86.16
47	81.44	80.50
48	77.83	96.05
49	76.79	87.61
50	80.64	94.68
51	80.78	83.35

**Table 3:** Statistical table of familiarity of patients' pathological knowledge.

No.	Control group	Test group
1	66.95	63.75
2	72.62	79.80
3	59.78	56.72
4	49.56	53.42
5	76.86	77.40
6	58.69	81.63
7	77.71	51.88
8	60.11	70.48
9	45.53	65.92
10	54.55	71.75
11	69.63	53.93
12	75.28	75.16
13	45.91	74.68
14	60.68	60.76
15	51.41	75.32
16	74.21	64.67
17	77.18	80.54
18	69.04	59.70
19	68.16	68.40
20	69.45	59.73
21	61.57	64.98
22	73.00	55.61
23	65.80	78.34
24	53.17	67.72
25	62.17	50.91
26	76.83	51.25
27	76.36	76.04
28	55.96	56.91
29	51.86	52.67
30	77.77	80.41
31	72.34	51.31
32	56.32	75.08
33	54.58	67.95
34	63.09	62.53
35	70.04	55.32
36	70.44	71.66
37	73.66	74.56
38	73.32	52.05
39	49.69	78.28
40	46.29	54.28
41	72.07	56.20
42	52.30	82.17
43	72.04	67.09
44	73.86	68.51
45	53.25	52.62
46	62.82	79.38
47	55.15	82.21
48	72.33	54.55
49	46.21	61.74
50	66.44	72.04
51	74.92	60.72

**Table 4:** Statistical table of the effect of patients' autonomous nursing.

No.	Control group	Test group
1	81.20	50.31
2	57.77	73.55
3	65.06	50.49
4	42.64	82.43
5	51.00	51.77
6	74.80	55.45
7	72.55	60.59
8	68.43	75.69
9	44.23	66.91
10	46.93	79.97
11	66.80	78.75
12	80.14	68.91
13	50.27	53.97
14	65.24	60.42
15	51.60	79.76
16	46.65	80.58
17	51.51	78.37
18	51.13	60.45
19	63.68	52.91
20	41.43	63.75
21	46.87	59.55
22	78.40	65.67
23	47.70	61.61
24	77.86	83.95
25	78.89	55.24
26	44.56	58.57
27	43.18	63.80
28	55.67	84.87
29	60.93	51.92
30	47.18	70.41
31	46.13	67.74
32	66.35	61.37
33	42.20	70.10
34	66.37	68.83
35	52.93	52.99
36	61.96	75.64
37	80.98	79.10
38	77.58	65.07
39	57.45	78.60
40	41.46	84.50
41	55.62	57.41
42	41.45	81.42
43	78.58	83.47
44	64.82	56.18
45	52.73	53.75
46	48.06	77.87
47	55.79	78.61
48	56.58	77.77
49	78.85	68.67
50	53.15	65.32
51	76.26	83.96

**Table 5:** Statistical table on the enthusiasm of patients and their families.

No.	Control group	Test group
1	80.05	88.90
2	86.68	76.21
3	70.97	78.32
4	66.02	75.09
5	60.68	83.70
6	87.55	85.74
7	88.83	86.67
8	63.77	81.37
9	74.65	80.04
10	90.22	91.61
11	72.04	82.14
12	76.53	92.93
13	78.41	80.27
14	84.23	91.72
15	81.48	78.90
16	83.20	75.22
17	63.19	90.94
18	61.52	74.05
19	86.53	80.84
20	73.60	76.86
21	84.22	90.17
22	66.33	85.46
23	86.65	94.55
24	61.66	88.60
25	89.91	93.67
26	75.93	81.05
27	76.69	74.67
28	70.07	94.09
29	64.83	87.08
30	71.77	81.15
31	74.61	80.58
32	89.66	78.51
33	81.85	88.47
34	89.90	90.24
35	72.60	90.98
36	86.77	91.63
37	77.92	80.44
38	65.95	75.84
39	76.39	88.25
40	85.46	83.82
41	56.32	83.34
42	78.45	80.96
43	82.69	88.21
44	69.31	76.76
45	80.91	93.02
46	71.45	90.30
47	82.60	81.36
48	76.89	80.94
49	55.88	91.66
50	86.00	76.90
51	68.01	93.43

## Data Availability

The data used to support the findings of this study are included within the article.
